# Copying and Recreation Methods of Painting Works Relying on Mobile Digital Multimedia Big Data Analysis

**DOI:** 10.1155/2022/7734506

**Published:** 2022-01-06

**Authors:** Li Xue, Chuangjian Yang

**Affiliations:** ^1^School of Arts, East China Jiaotong University, Nanchang 330013, China; ^2^School of Physical Education and Health, East China Jiaotong University, Nanchang 330013, China

## Abstract

In order to improve the effect of copying and recreation of painting works, this paper combines mobile digital multimedia big data technology to improve the image coding algorithm, identify the characteristics of existing works, apply the algorithm to the detailed analysis of painting works, and construct the main functional structure modules of the system. Moreover, this paper combines the existing hardware equipment to construct the painting works' recreation system and obtains the image processing module. After the system is constructed, the effect of copying and recreating painting works is analyzed through the mobile digital multimedia big data analysis technology. Finally, this paper constructs the system of this paper through simulation methods and uses experiments to calculate the feature recognition effect and copy effect of the painting works of the system. Through experimental analysis, it can be known that the copying and recreation system of painting works based on mobile digital multimedia big data analysis proposed in this paper can help painters effectively improve the effect of recreation.

## 1. Introduction

With the development of society and the progress of the times, mankind is increasingly inseparable from the efficiency and convenience brought by high technology. While it brings new changes to people's lives, it also brings a new art form to the art field, that is, digital technology. It is widely used and diversified in artistic expression methods. In today's technological era, it has an extremely broad development space [1]. The development of digital technology has expanded the way human beings live. In particular, the combination of digital technology and art has established a new type of visual language relationship based on easel painting, that is, a new relationship between humans-art-digital technology-digital art. This relationship boldly changed the way people observe and understand the art world and opened up a whole new space for people to explore the art world. In the long history of today's social development, science and art, like the two giant currents produced by human civilization, have gone through a variety of development processes of convergence and separation. The relationship between science and art has always been mutual promotion and coordinated development [2]. When digital art enters the era of Internet media communication, it has set off an unprecedented evolution for the development of art. In particular, it has had a profound impact and a huge impact on easel painting and has formed new changes. The changes include two major aspects: material and technological foundations and ideological concepts. In the art world, perhaps many artists once doubted and rejected the application value of computer technology. However, in the context of the development of today's globalized economy, the emergence of the “image age and visual feast” has broadened people's artistic vision and increased their demand for art. At present, the development of digital technology has been unstoppable, and many artists have gradually accepted the new changes made by modern digital technology to artistic creation and have begun to jointly explore new directions for the development of digital technology and easel painting [3].

Artists have their own unique ways of understanding, and sometimes, they even lead the entire society to re-examine the world. And works of art are not only the reproduction of the perception of space, whether it is Egyptian-style plane cognition or Renaissance-style cognition, they often have more complex and richer content pursuits. However, this inevitably makes the expression of art fall into a kind of contradiction: on the one hand, artists need to express their own feelings and emotional appeals, and they need to tell the spirit and stories of the times. This makes the picture must contain plot, concept, divinity, and humanity; poetry and even music are nonspatial content; on the other hand, their medium is often limited to a very limited canvas. So, two unavoidable questions arise: one is what space should be expressed, and the other is how to express the desired space.

The cutting-edge illustration of digital technology style is a combination of fashion elements and original concepts. In the development process of the times, it has been applied in various fields, penetrated into all aspects of life, and attracted more people's attention. Through in-depth research and generalization of this topic, people can have a more comprehensive and specific understanding of the visual characteristics, technical beauty, and artistic beauty of cutting-edge illustrations. The cutting-edge illustrations of digital technology style have attracted more and more people's attention and have played an important role in the process of the times.

This study combines mobile digital multimedia big data technology to carry out research on the copying and recreation of painting works and provides a reference for the development of intelligent computer technology in the direction of artistic creation.

## 2. Related Work

Google's Tilt Brush is an application that draws stereo images in a virtual space. To some extent, it has liberated human artistic creativity in a breakthrough. Tilt Brush is a VR application based on HTC Vive. A virtual environment is simulated by a computer to generate unlimited virtual painting space to replace the limited canvas [4]. Creators can create in three-dimensional space by wearing a VR helmet and using a controller that mimics painting gestures and can freely shuttle through the work while painting. For painting in three-dimensional space [5], the creator will directly interact with the three-dimensional model of the work, which replaces the previous procedural computer operation [6]. This will infinitely increase the degree of creative freedom, completely let go of the designer's thinking, and give the designer a brush for creative inspiration. The development of virtual reality and augmented reality technology is advancing by leaps and bounds, attracting more and more artists to enter the field of virtual space creation [7]. The virtual space painting brought about by virtual reality technology broke the previous situation where creators could only be limited to flat paper or software for painting creation [8]. Creating art in a three-dimensional space is a new way of thinking, which broadens the path of human creativity and opens the door to imagination. The literature [9] tried to use VR painting to create the Little Mermaid Ariel. There is no edge of the canvas in the virtual space. This has surpassed the traditional flat painting and developed into a sculpture creation. The revolution brought by VR painting not only is a breakthrough from two-dimensional to three-dimensional but can also change the creative process and method of painting by freely moving the position and perspective of the painter [10].

Virtual reality, or VR, for short, technology is a computer interactive three-dimensional dynamic visual scene and entity behavior simulation system that can create and experience virtual worlds [11]. VR devices include head-mounted display devices and control handles. By wearing a VR device, the user can be immersed in the virtual environment simulated by the device, giving the user an immersive feeling and a realistic experience effect [12]. Thanks to breakthroughs in computer hardware equipment, virtual reality (VR) and augmented reality (AR) technologies have developed rapidly and become popular, gradually spreading to applications in all walks of life [13]. The core concepts of VR painting are interactivity, immersion, and imagination. Immersion is a kind of deceptive subjective consciousness. The feeling of being completely in it is based on the audience's extremely high-precision tracking and adjustment of the visual and auditory perception through the VR device on the basis of the virtual environment. A similar illusion is discussed in [14]. Different from traditional paintings or computer digital paintings, when creators create VR paintings based on virtual reality systems, they can walk into the screens themselves, form a highly harmonious interaction with the works, and even become themselves part of the work. This strongest sense of immersion can easily inspire creators and realize their creativity easily [15].

## 3. Mobile Multimedia Big Data Image Coding

Encoding is a technique that converts analog modulated signals into digital signals. The image coding technology is not only the application of linear pulse code modulation (linear PCM) but also the use of the statistical characteristics of the image signal and the physiological and psychological characteristics of the image to encode the image.

The model shown in Figure 1 is a digital communication system model. In such a model, there are secondary coding and decoding, that is, source coding, source decoding, channel coding, and channel decoding. The main task of source coding is to solve the validity problem, that is, to compress the source to make the processed signal more suitable for the digital communication system.

A lossless predictive coding system is mainly composed of an encoder and a decoder, as shown in Figure 2. They each have the same predictor. When the pixel sequence *f*_*n*_ (*n* = 1,…) of the input image enters the encoder one by one, the predictor generates the predicted (estimated) value of the current input pixel according to a number of past inputs. The output of the predictor is rounded to the nearest integer *f*_*n*_′ and used to calculate the prediction error [16]:

(1) $$\begin{array}{c} e_{n}=f_{n}-f_{n}^{\prime }. \end{array}$$

This error is encoded by the symbol encoder with the help of variable-length codes to generate the next element of the compressed data stream. Then, the decoder reconstructs encoder according to the received variable-length codeword and performs the following operations:

(2) $$\begin{array}{c} f_{n}=f_{n}^{\prime }+e_{n}. \end{array}$$

In most cases, the prediction can be obtained by linearly combining *m* previous pixels [17]:

(3) $$\begin{array}{c} f_{n}=\text{round}\left[\sum_{i=1}^{n}a_{i}f_{n-1}\right], \end{array}$$

where *m* is the order of the linear predictor, round is the rounding function, and *a*_*i*_ is the prediction function. In 1-*D* linear predictive coding, the above formula can be written as

(4) $$\begin{array}{c} f_{n}=\text{round}\left[\sum_{i=1}^{n}a_{i}f_{n-1}\left(x,y-i\right)\right]. \end{array}$$

In encoding, prediction is a function of the previous pixels scanned when the image is scanned from left to right and from top to bottom. Moreover, it can be seen from the above formula that the first *m* pixels of each line cannot be predicted and calculated, so these pixels are coded in other ways. This is the extra cost of predictive coding, which needs to be considered when high dimensional.

The structural block diagram of the lossy predictive encoder is shown in Figure 3. It has one more quantization link than the lossless predictive encoder. The quantizer is set between the symbol encoding and the place where the prediction error is generated and absorbs the integer rounding module in the original lossless prediction encoder. At the same time, it maps the prediction error into a finite number of outputs *e*_*n*_′, which determine the amount of compression and distortion of the lossy prediction coding.

In the encoding process, the system has an additional feedback link, and its input is a function of past predictions and corresponding quantization errors:

(5) $$\begin{array}{c} {\hat{f}}_{n}=f_{n}^{\prime }+{\hat{e}}_{n}. \end{array}$$

The optimal predictor used in most predictive coding satisfies the constraints as follows [18]:

(6) $$\begin{array}{c} {\hat{f}}_{n}=f_{n}^{\prime }+{\hat{e}}_{n}\approx f_{n}^{\prime }+e_{n},\\ f_{n}^{\prime }=\sum_{i=1}^{m}a_{i}f_{n-i}. \end{array}$$

Under this condition, the mean square predictive coding of the encoder is minimized:

(7) $$\begin{array}{c} E\left\{e_{n}^{2}\right\}=E\left\{{\left[f_{n}-f_{n}^{\prime }\right]}^{2}\right\}=E\left\{{\left[f_{n}-\sum_{i=1}^{m}a_{i}f_{n-i}\right]}^{2}\right\}. \end{array}$$

Among them, the sum of coefficients is set to be less than or equal to 1, namely,

(8) $$\begin{array}{c} \sum_{i=1}^{m}a_{i}\leq 1. \end{array}$$

The optimization criterion here is to minimize the mean square error, and the design of the optimal predictor becomes a problem of selecting *m* prediction coefficients. The solution can be obtained by deriving each coefficient of the above formula to find the extreme value. Corresponding to different coefficients, different predictors will be obtained.

Information is defined as a measure of uncertainty. The less likely a message is, the more information it has. The greater the likelihood of a message, the smaller its information. Mathematically, the transmitted message is a monotonically decreasing function of its probability of occurrence. The so-called amount of information refers to the measurement or content of information needed to select an event from *N* equally possible events, that is, the minimum number of questions “yes or no” in the process of identifying a specific event among *N* events.

The probability of selecting any number *x* from *N* numbers is *p*(*x*). We assume that the probability of choosing any number is equal, that is, *p*(*x*) = 1/*N*, so the amount of information is defined as [19]

(9) $$\begin{array}{c} I\left(x\right)=\;\log_{2}\;N=-\log_{2}\;p\left(x\right)=I\left[p\left(x\right)\right]. \end{array}$$

If the information amount of all possible events of the source is averaged, the “entropy” of the information is obtained, and the entropy is the average amount of information. The symbol set of the source *X* is *x*_*i*_ (*i* = 1, 2,…, *N*), and the probability of occurrence is *p*(*x*_*i*_). Then, the information entropy of source *X* is

(10) $$\begin{array}{c} H\left(X\right)=\sum_{i=1}^{N}p\left(x_{i}\right)I\left[p\left(x_{i}\right)\right]=-\sum_{i=1}^{N}p\left(x_{i}\right)\log_{2}\;p\left(x_{i}\right). \end{array}$$

Information entropy has the following properties:

1. Entropy is a nonnegative number, that is, *H*(*x*) ≥ 0. When *P*(*x*) = 0 or *P*(*x*) = 1, *H*(*x*) = 0.
2. *H*(*x*) ≤ log_2_*M*, where *M* is the number of states of *x*. When *p*(*x*_*i*_)=1/*M*, the equal sign is established.
3. The joint entropy is *H*(*x*, *y*) ≤ *H*(*X*) + *H*(*Y*), and the equal sign holds when *X* and *Y* are independent.
4. The conditional entropy is *H*(*X|Y*)=*H*(*X*, *Y*) − *H*(*Y*) ≤ *H*(*X*), and the equal sign holds when *X* and *Y* count independently.

Line-level coding is a relatively simple type of coding, which refers to comparing the amplitude (such as brightness) of neighboring pixels among pixels scanned in a line. When there is a significant change in the amplitude, it means that there is a stroke. The continuous length of the pixel amplitude and the end position mark are its important parameters. Depending on the endpoint marking method, the stroke encoding can be divided into two categories:

(1) Stroke end code: the end position of the stroke is determined by the number of pixels from the start point of the scan line to the end position of the stroke.
(2) Stroke length coding: the end position of a certain stroke is determined by its relative distance from the previous end point. There are two types of end-of-stroke encoding.
  1. The linear code method (A code) assigns different code words according to different run lengths. The long codeword is long with a large stroke, and the codeword is short with a small stroke.
  2. For the digital method (B code), the length of the code word is proportional to the logarithm of the run length.

Run length coding is suitable for binary images. The efficiency of run length coding is not as high as that of Huffman coding, but its codeword structure is relatively simple, so it is also used in many cases.

Compared with DCT coding, the biggest advantage of subband coding is that the restored image has no block effect. Therefore, it has been extensively studied and is a promising image coding method. The statistical characteristics of each subband image are determined by the sensitivity of the human eye to them. According to the information theory and the visual characteristics of the human eye, different methods are used to encode each subband. The main points can be summarized as the following two points:

1. The LL component is the most important and should be encoded more accurately. Generally, DPCM, DCT, and other methods can be used, and the quantization should be more accurate.
2. The importance of high-frequency components is less important, and it is not suitable for DCT encoding. Since DPCM is not much better than PCM, it is usually directly encoded with PCM. In addition, in order to reduce the impact of code rate and noise, the quantization of high-frequency components has a dead zone near zero.

The theoretical basis of fractal image compression is the iterative function system IFS theorem, shrinkage mapping theorem, and collage theorem. An iterative function system consists of a complete metric space and a set of contraction maps on it. The contraction mapping theorem tells us that every convergent mapping in the function space has a fixed point. This makes the point sequence formed after each point in the function space undergoes the continuous action of this shrinkage map to converge to this fixed point. The iterative function system theorem states that every iterative function system can form a contraction map in the function space. In the decoding process, the iterative function system is determined by the corresponding parameters, and the image is generated through iteration according to the theorem of the iterative function system.

There are two basic methods for fractal image compression coding:

1. Manually intervened interactive fractal image coding method: it mainly uses traditional image processing techniques such as edge detection, spectrum analysis, texture analysis, and fractal method for image segmentation according to the shape of a given image. It requires that each part to be separated has relatively intuitive self-similar characteristics. Then, it looks for an iterative function system and determines each transformation system. Furthermore, it obtains the concomitant probability of each transformation from the grayscale distribution in the image. The decoding process uses a random iterative method to generate an approximate image. The compression ratio of this method is generally quite high.
2. Adaptive block fractal coding method: it first divides the image into several nonoverlapping range blocks *R*_*i*_ and overlapping domain blocks *D*_*i*_. Next, the algorithm finds a certain *R*_*i*_ for each *D*_*i*_ so that *D*_*j*_ is mapped to *R*_*j*_ through a certain specified transformation to achieve the specified minimum error and records the parameters to determine *R*_*j*_ and *D*_*j*_ and the transformation *w*_*j*_ to obtain an iterative function system. Finally, the algorithm encodes these parameters.

Whether in the time domain or in the frequency domain, a wavelet is a function that exists locally at a certain position, and its waveform only changes in amplitude at a certain position. Since the frequency is inversely proportional to the period, when the low-frequency component of the signal is to be analyzed, the basic wavelet can be amplified by a times. Conversely, when the high-frequency component of the signal is to be analyzed, it can be done by reducing *a* times. In addition, in order to find the time when the signal changes, you can move *b* seconds on the time axis to finally form the basis function. If *φ*(*t*) is used to represent the mother wavelet (basic wavelet), the basic wavelet construction bottom basis function *φ*_*a*,*b*_(*t*) should be [20]

(11) $$\begin{array}{c} \varphi_{a,b}\left(t\right)=\frac{1}{\sqrt{a}}\varphi \left(\frac{t-b}{a}\right). \end{array}$$

For a given signal *f*_0_, its wavelet transform can be defined as

(12) $$\begin{array}{c} W_{f}\left(a,b\right)=\langle f\left(t\right),\varphi_{a,b}\left(t\right)\rangle =\frac{1}{\sqrt{a}}\int_{R}f\left(t\right)\varphi^{*}\left(\frac{t-b}{a}\right). \end{array}$$

That is, the continuous function of *f*(*t*) can be regarded as the scalar product of *f*(*t*) and the two-parameter function *φ*_*a*,*b*_(*t*). At the same time, the mother wavelet must meet the following conditions:

(13) $$\begin{array}{c} \int_{-\infty }^{+\infty }\varphi \left(t\right)=0. \end{array}$$

If we assume

(14) $$\begin{array}{c} C_{\varphi }=\int_{-\infty }^{+\infty }\frac{{\left|\varphi \left(t\right)\right|}^{2}}{t}\text{d}t, \end{array}$$

then the reconstruction of *f*(*t*) can be expressed by the following formula [21]:

(15) $$\begin{array}{c} f\left(t\right)=C_{\varphi }^{-1}\int_{-\infty }^{+\infty }\int_{-\infty }^{+\infty }\varphi_{a,b}F\left(a,b\right)\text{d}bab\frac{\text{d}a}{a^{2}}. \end{array}$$

The main features of wavelet transform are

1. For high-frequency components, the resolution of time will be; for low-frequency components, the resolution of frequency will have the practical ability of multiresolution analysis.
2. The position of the waveform is a certain local position. Because there is no DC component, it is particularly sensitive to the changing points (discontinuities) of the waveform.
3. The size of the local function on the axis is local. Therefore, as long as *a* and *b* are sufficiently dense, a very stable signal sequence can be completely reconstructed.

The above analysis shows that, in a continuous situation, as long as both *a* and *b* are known, the original signal can be completely reconstructed. However, in practical applications, more discrete digital processing methods are used, and these parameters are limited to discrete grids. At this time, depending on the size of the grid, the information contained in the coefficients will be partially incomplete, and it will be difficult to fully realize the reconstruction. The function of continuous wavelet basis function in wavelet analysis and synthesis is just like an orthogonal basis. For the discretized wavelet transform, the discretization time-scale parameters *a* and *b* are appropriately selected to obtain a true orthogonal basis. When the parameters *a* and *b* are defined as

(16) $$\begin{array}{c} a=a_{0}^{m},\\ b=kb_{0}a_{0}^{n}, \end{array}$$

among them, *m* and *n* are integers, and the corresponding wavelet is

(17) $$\begin{array}{c} \varphi_{m,n}\left(t\right)=\varphi_{a_{0}^{w},kb_{0}a_{0}^{n}}\left(t\right)=a_{0}^{-m/2}\varphi \left(a_{0}^{-m}t-nb_{0}\right). \end{array}$$

The discrete wavelet transform of function *f* is redefined as

(18) $$\begin{array}{c} F\left(m,n\right)=\sum_{m,n}C_{m,n}\langle f,\varphi_{m,n}\rangle . \end{array}$$

Signal reconstruction is to find *a*_0_, *b*_0_, and *φ*(*t*) to make

(19) $$\begin{array}{c} f\left(t\right)\approx c\sum \sum C_{m,n}\varphi_{m,n}\left(t\right). \end{array}$$

*c* is a constant that has nothing to do with the signal. When *a*_0_ is close enough to 1, the wavelet function is over-complete, and the signal reconstruction is realized within the unrestricted range of *φ*_*a*,*b*_(*t*). On the contrary, if the sampling is sparse, a true orthogonal basis can only be obtained when a very special *φ*_*a*,*b*_(*t*) is selected.

**Definition 1 .**

We call a sequence of subspace {*V*_*j*_}_*j*∈*z*_ and a function *φ*(*t*) in *L*^2^(*R*) satisfying the following conditions as an orthogonal multiscale analysis, denoted as ({*V*_*j*_}_*j*∈*z*_, *φ*(*t*)):

1. *V*_*j*_ ⊆ *V*_*j*−1_, *j* ∈ *z*
2. *f*(*t*) ⊆ *V*_*j*_ ⟺ *f*(2*t*) ∈ *V*_*j*−1_
3. ∩_*j*∈*z*_*V*_*j*_={0}, ∩_*j*∈*z*_*V*_*i*_=*L*^2^(*R*)
4. *φ*(*t*) ∈ *V*_0_, and {*φ*(*t* − *k*)}_*k*∈*z*_ is the orthonormal basis of *V*_0_, and *φ*(*t*) is the scaling function or parent function of this multiscale analysis

From properties (2) and (4), we know that, for any *f*(*t*) ∈ *V*_0_, there is *f*(*t*/2^*j*^) ∈ *V*_*j*_ and it is easy to verify. The function system {2^−*j*/2^*φ*(2^−*j*^*t* − *k*)}_*k*∈*z*_ constitutes a set of standard orthogonal basis of *V*_0_.

Since *V*_*j*_ ⊆ *V*_*j*−1_, *W*_*j*_ is the orthogonal complement space of *V*_*j*_ in *V*_*j*−1_, that is, *V*_*j*−1_=*V*_*j*_+*W*_*j*_, *V*_*j*_ ⊥ *W*_*j*_, *j* ∈ *z*. In this way, the space column {*W*_*j*_}_*j*∈*z*_ is obtained. Obviously, when *m*, *n* ∈ *z* and *m* ≠ *n*, there is *W*_*m*_ ⊥ *W*_*n*_. In addition,

(20) $$\begin{array}{c} V_{j-1}=V_{j}+W_{j}=V_{j+1}+W_{j+1}+W_{j+1}\\ =V_{j+2}+W_{j+2}+W_{j+1}+W_{j}=\cdots \\ =V_{j+1}+W_{j+s}+W_{j+s-1}+\cdots +W_{j+1}+W_{j}. \end{array}$$

When *s*⟶+*∞*, we obtain

(21) $$\begin{array}{c} V_{j-1}=\overset{+\infty }{\underset{m=j}{⊕}}W_{m}. \end{array}$$

When *s*⟶−*∞*, we obtain

(22) $$\begin{array}{c} V_{j-1}=\overset{+\infty }{\underset{m=-\infty }{⊕}}W_{m}. \end{array}$$

We also call *W*_*j*_ the wavelet space with scale *j* and *V*_*j*_ the scale space with scale *j*. Since *W*_*j*_ is the orthogonal complement of *V*_*j*_ in *V*_*j*−1_, *W*_*j*_ is also called the detail space of *V*_*j*_ in *V*_*j*−1_.

In this way, the approximation of a signal *f*(*t*) at resolution 2^−*j*^ defines its orthogonal projection on space *V*_*j*_ ⊂ *L*^2^(*R*), and space *V*_*j*_ gathers all possible approximations at resolution 2^−*j*^.

The basic function of a two-dimensional wavelet transform can be obtained:

(23) $$\begin{array}{c} \varphi^{1}\left(x,y\right)=\phi \left(x\right)\varphi \left(y\right),\\ \varphi^{2}\left(x,y\right)=\phi \left(x\right)\varphi \left(y\right),\\ \varphi^{2}\left(x,y\right)=\phi \left(x\right)\varphi \left(y\right). \end{array}$$

The image can be regarded as a two-dimensional matrix. Generally, it is assumed that the size of the image matrix is *N* × *N* and *N* = 2*n* (*n* is a nonnegative integer). Then, after each wavelet transformation, the image is decomposed into 4 subblock frequency band regions whose size is 1/4 of the original size, as shown in Figure 4. The wavelet coefficients of the corresponding frequency bands are included, respectively, which is equivalent to sampling at intervals in the horizontal and vertical directions. When the next wavelet transform is performed, the transformed data are concentrated in the LL frequency band.  Figure 5 shows the coefficient distribution of the three-layer wavelet transform.

The following equation illustrates the mathematical model of image wavelet transform.

LL frequency band: this frequency band retains the content information of the original image, and the energy of the image is concentrated in this frequency band:
  (24) $$\begin{array}{c} f_{2^{j}}^{0}\left(m,n\right)=\langle f_{2^{j-1}}\left(x,y\right),\phi \left(x-2m,y-2n\right)\rangle . \end{array}$$
HL frequency band: this frequency band maintains high-frequency edge information in the horizontal direction of the image:
  (25) $$\begin{array}{c} f_{2^{j}}^{1}\left(m,n\right)=\langle f_{2^{j-1}}\left(x,y\right),\varphi^{1}\left(x-2m,y-2n\right)\rangle . \end{array}$$
LH band: this frequency maintains the high-frequency edge information in the vertical direction of the image:
  (26) $$\begin{array}{c} f_{2^{j}}^{2}\left(m,n\right)=\langle f_{2^{j-1}}\left(x,y\right),\varphi^{2}\left(x-2m,y-2n\right)\rangle . \end{array}$$
HH band: this band maintains the high-frequency edge information in the diagonal direction of the image:

(27) $$\begin{array}{c} f_{2^{j}}^{3}\left(m,n\right)=\langle f_{2^{j-1}}\left(x,y\right),\varphi^{3}\left(x-2m,y-2n\right)\rangle . \end{array}$$

Among them, 〈〉 〈〉 represents the inner product operation.

## 4. Copying and Recreation System of Painting Works Based on Mobile Digital Multimedia Big Data Analysis

The system structure is shown in Figure 6. The model contains several basic components. (1) Camera: one or more cameras are used to pick up visual information in the physical environment, that is, to pick up paints for paintings. (2) Image processing: it performs certain processing on the paints obtained by the camera. (3) Drawing module: it arranges the processed paint on the bottom of the painting. (4) The bottom of the painting: it carries the paint to form a painting and can update the content of the painting to the user in real time. (5) Interaction: it provides some control mechanisms that allow users to manipulate the camera, image processing, and interaction mechanisms.

The conceptual framework of the real-time video media painting tool is shown in Figure 7. It adopts a method similar to Glowdoodleu; its camera adopts an ordinary camera, and the image processing, drawing module, painting background, and interaction are all realized by computer programs. Its content is presented to the user in the form of a graphical interactive interface on the basic I/O device (input device).

The basic function of the image processing module is to process the RGB color image *F* input by the camera and to input the RGB color image *C* and the gray image *F* to the drawing module. Its internal operation is formed by combining multiple submodules. These modules include color-to-gray module, gray-to-color module, differential module, fixed image output module, color transmission module, deformation module, weighting module, and color adjustment module. The basic function of each module is to process the input image and output an image, as shown in Figure 8.

After constructing the above model, the copying and recreation system of painting works based on mobile digital multimedia big data analysis constructed in this paper is tested and analyzed, and the feature recognition effect and copy effect of the detection system are tested, and the results are shown in Figure 9.

From the above statistical analysis, it can be seen that the copying and recreation system of painting works based on mobile digital multimedia big data analysis proposed in this paper has a good performance in the feature recognition and copying of painting works. On this basis, this paper evaluates the recreation effect of the system constructed in this paper, and the results are shown in Figure 10.

From the above research, it can be seen that the copying and recreation system of painting works based on mobile digital multimedia big data analysis proposed in this paper can help painters effectively improve the recreation effect.

## 5. Conclusion

In digital painting, the creator can describe the dream state in his mind and enter the virtual space that belongs to him only. In traditional painting, due to the limitations of creative materials and creative methods, we cannot completely express the true form of three-dimensional objects on a flat canvas. What we can do is to choose and process the visible part of the object according to the perspective principle, and such works will inevitably have incompleteness from a three-dimensional perspective. However, the emergence of digital painting allows us to walk through paintings at will, appreciate them at any position and from any angle, and continuously improve our paintings. In the digital world, viewers can enter a colorful, full, flowing, and lively surreal world and experience the real touch surrounded by colors and lines. This article combines mobile digital multimedia big data technology to carry out research on copying and recreating painting works. In addition, this paper constructs an intelligent painting copying and recreation system and verifies the performance of the system. From the research, it can be seen that the method proposed in this paper has good results.

## Figures and Tables

**Figure 1:** Communication system model.

**Figure 2:** Lossless predictive coding system.

**Figure 3:** Lossy precoding system.

**Figure 4:** A high-dispersion wavelet transform.

**Figure 5:** Three-layer wavelet transform.

**Figure 6:** Copying and recreation system of painting works based on mobile digital multimedia big data analysis.

**Figure 7:** System conceptual model.

**Figure 8:** The components of the image processing module.

**Figure 9:** The feature recognition effect and copying effect of the system.

**Figure 10:** Evaluation of the recreation effect of the system.

## Data Availability

The labeled dataset used to support the findings of this study are available from the corresponding author upon request.
